The article "HDAC1-Mediated MicroRNA-124-5p Regulates NPY to Affect Learning and Memory Abilities in Rats with Depression" was retracted in 2023. Reasons: manipulated images; original data or images not available; unreliable results or conclusions; concerns about the images.

# HDAC1-Mediated MicroRNA-124-5p Regulates NPY to Affect Learning and Memory Abilities in Rats with Depression

**DOI:** 10.1186/s11671-021-03477-3

**Published:** 2021-02-10

**Authors:** Chunling Tang, Jian Hu

**Affiliations:** Department of Psychiatry, The First Affiliated Hospital of Harbin Medical University, 23 Youzheng Street, Nangang District, Harbin, 150001 Heilongjiang China

**Keywords:** Depression, Histone deacetylase 1, Neuropeptide Y, Learning, Memory

## Abstract

Researches pivoting on histone deacetylases (HDACs) in depression have been excessively conducted, but not much on HDAC1. Therein, the present study is launched to disclose the mechanism of HDAC1/microRNA (miR)-124-5p/neuropeptide Y (NPY) axis in depression. Sprague Dawley rats were stimulated by chronic unpredictable mild stress to establish depression models. Depressed rats were injected with inhibited HDAC1 or suppressed miR-124-5p to explore their roles in body weight, learning and memory abilities, oxidative stress and inflammation in serum and neurotransmitter expression in hippocampal tissues. MiR-124-5p, HDAC1 and NPY expression in the hippocampus were tested. The interactions of miR-124-5p, HDAC1 and NPY expression were also confirmed. Higher miR-124-5p and HDAC1 and lower NPY expression levels were found in the hippocampus of depressed rats. Inhibited miR-124-5p or suppressed HDAC1 attenuated learning and memory abilities and increased body weight of depressed rats. Knockdown of miR-124-5p or inhibition of HDAC1 suppressed oxidative stress and inflammation and promoted neurotransmitter expression of depressed rats. HDAC1 mediated miR-124-5p to regulate NPY. Knockdown of NPY abolished the protective effects of inhibited miR-124-5p on depressed rats. Our study illustrates that suppression of either miR-124-5p or HDAC1 up-regulates NPY to improve memory and learning abilities in depressed mice, which may update the existed knowledge of depression and provide a novel reference for treatment of depression.

## Introduction

Depression refers to a severe disabling psychosis that causes severe economic burdens and social consequences globally [1]. Depression is characterized by physiological, cognitive and behavioral changes that threatens patients’ overall health [2]. The treatments accessible to depression have developed with the application of ketamine as a fast-acting antidepressant and the refinement of equipment capable of selectively catering to the activity of populations of neuronal subtypes [3]. Moreover, versatile nanoarchitectures such as carbon dots are applicable for neurological disorders [4]. However, inadequate treatment for depression can results in poor performance, behavior dysfunctions, physical diseases, substance abuse and even suicide [5]. Thus, there is a desperate need to discover innovative agents in the treatment of depression.

The article "HDAC1-Mediated MicroRNA-124-5p Regulates NPY to Affect Learning and Memory Abilities in Rats with Depression" was retracted in 2023. Reasons: manipulated images; original data or images not available; unreliable results or conclusions; concerns about the images.

It is previously documented that microRNA (miR)-124 level raises in plasma with depression and antidepressants [6]. During chronic unpredictable mild stress (CUMS)-induced depression, miR-124 expression in the hippocampus shows dynamic variations, indicating various pathological changes at different stages of depression [7]. In addition, miR-124 is the candidate to ameliorate depressive-like behaviors in major depressive disorder [8]. Also, miR-124 suppression serves as an antidepressant in the prefrontal cortex, as reflected by attenuated depression-like behaviors in mice [9]. Histone deacetylase 1 (HDAC1) is a mediator of miR-124 [10] that forms a multi-protein complex for transcriptional regulation and epigenetic modification [11]. To our best knowledge, an impairment of HDAC1 activity promotes resilience in major depressive disorder [12]. Moreover, suppression of HDAC1 in the brain can improve mood disorders and other neuroplastically altered brain diseases [13]. HDAC inhibitors could attenuate anxiety-like and alcohol-drinking behaviors, and can elevate neuropeptide Y (NPY) expression [14]. Also, HDAC activity impairment can lead to an increase in the NPY expression in the central nucleus of amygdala and medial nucleus of amygdala [15]. NPY is a hypothalamic orexigenic neuropeptide which is sufficient to prevent anxiety, social disorders and depressive symptoms [16]. Besides that, NPY and its receptors have been evidenced to impose anti-inflammatory and antidepressant effects on lipopolysaccharides-induced depression rat models [17]. Taken together, the combined interplay of HDAC1/miR-124-5p/NPY axis in depression is in ambiguity. Thus, this study intends to unearth the mechanism of this axis to investigate a curative candidate for depression therapy.

## Materials and Methods

### Ethics Statement

The animal experiments involved in this study were adhered to the requirements of experimental animal ethics of The First Affiliated Hospital of Harbin Medical University. The experiments were optimized to improve experimental animal feeding conditions, reduce the number of animals used, and alleviate animal suffering.

### Experimental Animals

Sprague–Dawley (SD) male rats of specific pathogen-free (SPF) grade, weighing 200–220 g, were provided by the Animal Research Center, First Affiliated Hospital of Harbin Medical University (Harbin, China). The rats were kept in a SPF-grade environment (22–24 °C, 60–64% humidity, 12-h light and dark cycles). Except for the period during modeling and other specific time points, the rats were free to get water and food.

The article "HDAC1-Mediated MicroRNA-124-5p Regulates NPY to Affect Learning and Memory Abilities in Rats with Depression" was retracted in 2023. Reasons: manipulated images; original data or images not available; unreliable results or conclusions; concerns about the images.

### Rat grouping and Model Establishment

The modeled rats were randomly divided into 8 groups (*n* = 10): normal group (rats without any treatment), CUMS group (CUMS-induced depression rats), sh-negative control (NC) group (CUMS-induced depression rats injected with sh-HDAC1 lentivirus NC), sh-HDAC1 group (CUMS-induced depression rats injected with sh-HDAC1 lentivirus), anti-miR-NC group (CUMS-induced depression rats injected with anti-miR-124-5p lentivirus NC), anti-miR-124-5p group (CUMS-induced depression rats injected with anti-miR-124-5p lentivirus), anti-miR-124-5p + sh-NC group (CUMS-induced depression rats injected with anti-miR-124-5p lentivirus and sh-NPY lentivirus NC), and anti-miR-124-5p + sh-NPY group (CUMS-induced depression rats injected with anti-miR-124-5p lentivirus and sh-NPY lentivirus).

CUMS-induced depression rat models were established by Willner’s method [18]. The rats in the normal group were fed with food and water without any stimuli while rats in the other 7 groups received 35-days CUMS in independent cages. These rats were stimulated by ice-water swimming at 4 °C for 5 min in a container (30 cm of water depth), day and night inversion (rats staying in the dark for 12 h during the day and in a bright space illuminated by incandescent lamps for 12 h during the night), tail clamping by a swallow tail clip for 30 s, 1-min shaking, 24-h fasting and water deprivation, 30-min ultrasonic stimulation (50 Hz), wet padding, and air conditioning at 17℃. Rats were randomly stimulated by one of these stimuli daily, and the same stimulus was applied no more than 5 times in total.

Rats were anesthetized with 2% pentobarbital sodium (50 mg/kg) and bilateral hippocampus (anteroposterior diameter = 4.8 mm, mediolateral distance =  ± 2.5 mm, distance between back-cavity and anterior fontanelle = − 3.5 mm) were injected with lentivirus at 1 μL/min by a Hamilton micro-syringe with a 26-G needle. The needle was kept in the injection site for 5 min to prevent reflux. The skulls were sealed with bone wax and the incisions were sutured, and the rats were recovered for 7 days [19]. sh-HDAC1 lentivirus and its NC, anti-miR-124-5p lentivirus and its NC, as well as sh-NPY and its NC (titer: 10^8^ TU/mL) were bought from GenePharma Co. Ltd. (Shanghai, China).

### Behavioral Function Tests

Rats were weighed on the day before CUMS modeling (on the 0 day), after CUMS modeling (on the 36th days), and after lentivirus interference (on the 52nd days).

Open field test (OFT) could detect the autonomic and exploratory behaviors of rats in a new environment, which was commonly used to evaluate depressive behaviors. This test was carried out in a black wooden open field box (100 cm × 100 cm × 50 cm) with a video tracking system placed above the open field box to record rat activities. The bottom of the open box was divided into 25 grids (20 cm × 20 cm) with white lines. The rats were placed in the central grid in a pre-defined random order and the amount of crossing the grid (rats entering a grid with limbs or double forelimbs with one hind limb) and incidence of rearing (rats lifting forelimbs and standing upright with one hind limb) were record by the video tracking system. This test was performed in a quiet and dim indoor environment. After every test, the open field box was cleaned with 75% alcohol to remove odors.

The article "HDAC1-Mediated MicroRNA-124-5p Regulates NPY to Affect Learning and Memory Abilities in Rats with Depression" was retracted in 2023. Reasons: manipulated images; original data or images not available; unreliable results or conclusions; concerns about the images.

Anhedonia was one of the crucial symptoms of depression. The sucrose preference test (SPT) could evaluate the depressive-like behaviors of rats. Before SPT, each rat was provided with 2 bottles of sugar water (1% sucrose, w/w) for 24 h, and with 1 bottle of sterile water and 1 bottle of sugar water for another 24 h. After that, sucrose preference percentage (SPP) of rats was detected as following: after 23-h fasting and water deprivation, rats were allowed to 1 bottle of sterile water and 1 bottle of sugar water (1% sucrose) for 30 min. After 1 h, the location of the two bottles was inverted and rats were free to these two bottles for another 30 min. During this 1 h, the consumption (mL) of these two bottles of sterile water and sugar water (1% sucrose) was measured and SPP was calculated. SPP = sugar water consumption/(sugar water consumption + sterile water consumption) × 100%.

Morris water maze test (MWM) was widely applied to evaluate the spatial learning and memory abilities of rats. MWM test was performed in a circular water tank (150 cm in diameter and 60 cm in height) with water depth of 40 cm. The water temperature was maintained at 22 ± 1 °C and the water was dyed into black with non-toxic and easy-to-clean dye. The tank and water surface were divided into 4 quadrants (SE, SW, NW and NE quadrants) with each quadrant decorated with its corresponding icon with bright color and special shape on the inner wall. The target platform was a circular transparent platform (11 cm in diameter), located at the center of the NE quadrant and immersed 1.5 cm below the water surface. A video tracking system was installed above the center of the tank to record the swimming speed, path, and the time spent on rats getting into the target platform and swimming in quadrants. Rats were placed into water from 4 quadrants in a random order and they were allowed to explore and board the target platform within 60 s. The time taken by rats to board the platform was recorded as the escape latency. If rats failed to board the target platform within 60 s, they were guided and the escape latency was recorded as 60 s. After each test, rats were allowed to stay on the target platform for 15 s and rats were trained 4 times a day for 5 days. The final escape latency was the average of the escape latency on the 3rd-5th. On the 6th days of the MWM test, space exploration test was performed. The target platform was removed from the water tank, and the rats entered the water from the SW quadrant. The time of rats swimming in the NE quadrant within 60 s was recorded as the space exploration time.

The article "HDAC1-Mediated MicroRNA-124-5p Regulates NPY to Affect Learning and Memory Abilities in Rats with Depression" was retracted in 2023. Reasons: manipulated images; original data or images not available; unreliable results or conclusions; concerns about the images.

Timeline of this experiment is shown in Fig. 1.

**Fig. 1:** Chronology of the present study

### Specimen Collection

One day after the last MWM test, the rats were euthanized and intraperitoneally injected with 2% pentobarbital sodium (50 mg/kg). The thoracic cavity was opened to obtain heart blood with a syringe, which was centrifuged 3 times at 3500 r/min for 15 min, and the supernatant was stored at − 20 °C. After blood collection, a catheter was inserted from the left ventricle to the aorta, and 500 mL normal saline was perfused to flush the whole blood. Hippocampal tissues were separated and placed in 1.5-mL centrifuge tubes, weighed and stored at − 80 °C. A part of the hippocampus was fixed with 4% paraformaldehyde for 2 h, dehydrated with gradient sucrose and embedded in paraffin.

### Oxidative Stress-Related and Inflammatory Index Detection

The serum was rewarmed for detection of superoxide dismutase (SOD), malondialchehyche (MDA), glutathione (GSH), interleukin(IL)-β, tumor necrosis factor-α (TNF-α), and nitric oxide (NO) concentration. Kits for detection of SOD, MDA and GSH were provided by Beyotime Institute of Biotechnology (Shanghai, China), while enzyme-linked immunosorbent assay (ELISA) kits for detection of IL-β, TNF-α and NO by NanJing JianCheng Bioengineering Institute (Nanjing, China).

### Hematoxylin–Eosin (HE) Staining

The paraffin sections were dewaxed, hydrated with ethanol, rinsed with distilled water and stained with hematoxylin staining solution for 20 min. After that, the sections were rinsed with tap water until the sections turned blue. Then, the sections were placed in 1% ethanolic hydrochloric acid solution for 10 s, rinsed with tap water and dehydrated with ethanol, which was followed by staining in eosin for 2 min, dehydration with high-concentration alcohol and permeabilization in xylene. Finally, the sections were sealed and observed under a biological microscope.

### Neurotransmitter Expression Detection

The hippocampal tissues were weighed and homogenized by ultrasound in normal saline (100 μL/10 mg). The homogenate was kept at 4 °C for 30 min, centrifuged at 12,000 rpm (4 °C) for 3 min to collect the supernatant. The protein concentration of the supernatant was detected by bicinchoninic acid (BCA) protein detection kit (CWBIO, Beijing, China) and the expression levels of norepinephrine (NE), serotonin (5-HT), and dopamine (DA) by ELISA kits. NE, 5-HT and DA ELISA kits were provided by Liweiping Biotechnology Co., Ltd. (Beijing, China).

The article "HDAC1-Mediated MicroRNA-124-5p Regulates NPY to Affect Learning and Memory Abilities in Rats with Depression" was retracted in 2023. Reasons: manipulated images; original data or images not available; unreliable results or conclusions; concerns about the images.

### Reverse transcription Quantitative Polymerase Chain Reaction (RT-qPCR)

RNA was extracted from hippocampal tissues by RNA extraction kit (Promega, Madison, WI, USA), and the concentration and purity of the RNA were detected by an ultraviolet spectrophotometer. Followed by the reverse transcription kit instructions (DRR047S, Takara, Dalian, China), RNA reverse transcription into complementary DNA (cDNA) was performed. mRNA was reversely transcribed into cDNA by GoldScript one-step RT-PCR Kit (Applied Biosystems, Carlsbad, CA, USA) while miRNA by Hairpin-it™ miRNA quantitative detection kit (GenePharma). RT-qPCR detection kit (Promega) was applied to detect HDAC1, miR-124-5p and NPY expression in tissues. U6 was indicated as an internal control for miR-124-5p while β-actin for HDAC1 and NPY. PCR primers were obtained from Sangon Biotech Co., Ltd. (Shanghai, China) (Table 1). The relative expression of target genes was calculated by 2^−△△^Ct method.

**Table 1:** Primer sequence

Gene	Primer sequence (5′-3′)
HDAC1	Forward: 5′-CATGCCAAGTGTGTGGAGTTCGT-3’
	Reverse: 5′-GTCCAGCACCGAGCGACATT-3’
miR-124-5p	Forward: 5′-TAAGGCACGCGGTGAATG-3’
	Reverse: 5′-GTGCAGGGTCCGAGGT-3’
NPY	Forward: 5′-TGTTTGGGCATTCTGGCTGAGG-3’
	Reverse: 5′-TTCTGGGGGCGTTTTCTGTGCT-3’
U6	Forward: 5′-TGGCCCCTGCGCAAGGATG-3’
	Reverse: 5′-AACGCTTCACGAATTTGCGT-3’
β-actin	Forward: 5′-CAATGAGCTGCGTGTGGC-3’
	Reverse: 5′ -GGGTCATCTTTTCACGGTTGG-3’

HDAC1, Histone deacetylase 1; miR-124-5p, microRNA-124-5p; NPY, Neuropeptide Y

### Western Blot Analysis

The hippocampal tissues were cut into pieces on ice and lysed by radio-immunoprecipitation assay lysate (Beijing Solarbio Science & Technology Co. Ltd., Beijing, China) to extract protein. The protein concentration was determined by BCA method. Total protein (50 μg) was added with 5 × sodium dodecyl sulfate (SDS) loading buffer at 1:4 and heated in a boiling water bath for 5 min. Then, the protein was subjected to sodium dodecyl sulphate polyacrylamide gel electrophoresis, electroblotted onto a membrane and blocked with 5% milk for 1 h. After that, the protein was probed with the primary antibodies against HDAC1 (1:1000, Cell Signaling Technology, Beverly, MA, USA), NPY (1:800, NeoMakers, Fremont, California, USA) and β-actin (1:1000, Abcam, Cambridge, MA, UK) overnight, and reprobed with horseradish peroxidase-labeled secondary antibody. The membrane was developed by enhanced chemiluminescence, and the optical density was calculated by Quantity One gray analysis software. The protein expression of the target gene was expressed as the ratio of the gray value to β-actin gray value.

The article "HDAC1-Mediated MicroRNA-124-5p Regulates NPY to Affect Learning and Memory Abilities in Rats with Depression" was retracted in 2023. Reasons: manipulated images; original data or images not available; unreliable results or conclusions; concerns about the images.

### Chromatin Immunoprecipitation (ChIP) Assay

ChIP assay was performed in conformity to the instructions of the EZ-ChIP kit (Millipore, Bedford, MA, USA). HEK293T cells were incubated with 1% formaldehyde for 10 min and terminated by glycine. Then, the cells were centrifuged at 2000 rpm for 5 min, and added with SDS Lysis Buffer for ultrasonication. Centrifuged at 10,000 g at 4℃ for 10 min, the cells (100 μL) were reacted with 900 μL ChIP Dilution Buffer, 20 μL of 50 × PIC and 60 μL ProteinA Agarose/Salmon Sperm DNA at 4℃ for 1 h, and were allowed to stand for 10 min. The precipitates were centrifuged at 700 rpm for 1 min with 20 μL as input. A tube was added with HDAC1 antibody (1 μL) and immunoglobulin G antibody and the other tube was added without antibody. The samples in the two tubes were incubated overnight, eluted and de-crosslinked. After DNA retrieval, the sample was tested by RT-qPCR.

### Dual Luciferase Reporter Gene Assay

Bioinformatics website (https://cm.jefferson.edu/rna22/Precomputed/) analyzed the binding sites of miR-124-5p and NPY. NPY-wild type (WT) and NPY-mutant (MUT) plasmids were generated by Huayueyang Biotechnology Co., Ltd. (Beijing, China). Combined with mimic NC or miR-124-5p mimic, the plasmids were transfected into HEK293T cells. Cell luciferase activity was determined by the luciferase detection kit (BioVision) and Glomax20/20 luminometer (Promega).

### Statistical Analysis

SPSS 21.0 statistical software (IBM Corp. Armonk, NY, USA) was utilized for data analysis. The results were expressed as mean ± standard deviation. Comparisons between two groups were tested by *t* test. Comparisons among multiple groups were evaluated by one-way analysis of variance (ANOVA), after which pairwise comparisons by Tukey’s post hoc test. *P* represented two-sided tests and *P* < 0.05 was considered of statistical significance.

## Results

### Inhibition of Either HDAC1 or miR-124-5p Increases the Weight of Depressed Rats

Rats were weighed 1 day before CUMS modeling (day 0), 1 day after cessation of modeling (day 36), and 7 days after lentivirus interference (day 52). No difference was detected in the body weight of rats in each group before modeling (all *P* > 0.05). After modeling, the rat weight decreased in the CUMS group, sh-NC group, sh-HDAC1 group, anti-miR-NC group and anti-miR-124-5p group versus the normal group (all *P* < 0.05). No discrepancy was noticed as to rat weight in the CUMS group, sh-NC group, sh-HDAC1 group, anti-miR-NC group and anti-miR-124-5p group (all *P* > 0.05). After interference, the rat weight decreased in the CUMS group versus the normal group (all *P* < 0.05). No discrepancy was noticed as to rat weight in the CUMS group, sh-NC group, and anti-miR-NC group (all *P* > 0.05). The rat weight increased in sh-HDAC1 group and anti-miR-124-5p group relative to their NC groups (both *P* < 0.05), indicating that inhibition of HDAC1 or miR-124-5p increased weight of depressed rats (Fig. 2a).

The article "HDAC1-Mediated MicroRNA-124-5p Regulates NPY to Affect Learning and Memory Abilities in Rats with Depression" was retracted in 2023. Reasons: manipulated images; original data or images not available; unreliable results or conclusions; concerns about the images.

**Fig. 2:** Inhibition of either HDAC1 or miR-124-5p increases weight and improves learning and memory abilities of depressed rats. **a** Effects of inhibition with HDAC1 or miR-124-5p on the body weight of depressed rats; **b** SPP before and after inhibition with HDAC1 or miR-124-5p; **c** Frequency of crossing the gird in OFT before and after inhibition with HDAC1 or miR-124-5p; **d** Incidence of rearing in OFT before and after inhibition with HDAC1 or miR-124-5p; **e** Escape latency in MWM test before and after inhibition with HDAC1 or miR-124-5p; **f** Space exploration time in MWM test before and after inhibition with HDAC1 or miR-124-5p; *n* = 10; a *P* < 0.05 compared with the normal group; b *P* < 0.05 compared with the sh-NC group; c *P* < 0.05 compared with the anti-miR-NC group. Comparisons among multiple groups were evaluated by one-way ANOVA, and pairwise comparisons by Tukey’s post hoc test

### Inhibition of EITHER HDAC1 or miR-124-5p Improves Learning and Memory Abilities in Depressed Rats

SPT, OFT and MWM test were applied to detect SPP, frequency of crossing the grid and incidence of rearing, as well as escape latency and space exploration time. It was outlined that (Fig. 2b–f) before interference, in comparison with the normal group, SPP, frequency of crossing the grid, incidence of rearing and space exploration time reduced, whereas escape latency prolonged in the CUMS group, sh-NC group, sh-HDAC1 group, anti-miR-NC group and anti-miR-124-5p group (all *P* < 0.05), suggesting the development of depression-like behaviors in rats. There was no discrepancy in SPP, frequency of crossing the grid, incidence of rearing, space exploration time and escape latency among the CUMS group, sh-NC group, sh-HDAC1 group, anti-miR-NC group and anti-miR-124-5p group (all *P* > 0.05). After interference, versus the sh-NC group and anti-miR-NC group, SPP, frequency of crossing the grid, incidence of rearing and space exploration time increased while escape latency shortened in the sh-HDAC1 group and anti-miR-124-5p group (all *P* < 0.05). No difference was observed in SPP, frequency of crossing the grid, incidence of rearing, space exploration time and escape latency among the CUMS group, sh-NC group and anti-miR-NC group (all *P* > 0.05), suggesting that silencing of HDAC1 or suppression of miR-124-5p could attenuate depression-like behaviors and improve learning and memory abilities in rats.

The article "HDAC1-Mediated MicroRNA-124-5p Regulates NPY to Affect Learning and Memory Abilities in Rats with Depression" was retracted in 2023. Reasons: manipulated images; original data or images not available; unreliable results or conclusions; concerns about the images.

### Inhibition of Either HDAC1 or miR-124-5p Attenuates Pathological Neuron Damage in Depressed Rats

Observation of hippocampal lesions by HE staining (Fig. 3a) revealed that the neatly arranged neurons in the hippocampus of rats in the normal group showed clear morphology, normal structure, dense layers, clear cell nuclei, and obvious nucleoli. The neurons of rats in the CUMS group were shrunk, decreased in number and loosely arranged with unevenly distributed chromatin and thinned layer. The rats in the sh-NC and anti-miR-NC groups showed the same situation as the CUMS group. The rats in the sh-HDAC1 and anti-miR-124-5p groups displayed increased neurons in order and attenuated damage by comparison with their NC groups. It was indicated that knockdown of HDAC1 or inhibition of miR-124-5p alleviated hippocampal lesions in depressed rats.

**Fig. 3:** Inhibition of either HDAC1 or miR-124-5p attenuates pathological hippocampus damage and up-regulates neurotransmitter expression in depressed rats. **a** HE staining of hippocampal lesions of depressed rats; **b** ELISA of NE expression in hippocampal tissues; **c** ELISA of 5-HT expression in hippocampal tissues; **d** ELISA of DA expression in hippocampal tissues; *n* = 6; a *P* < 0.05 compared with the normal group; b *P* < 0.05 compared with the sh-NC group; c *P* < 0.05 compared with the anti-miR-NC group. Comparisons among multiple groups were evaluated by one-way ANOVA, and pairwise comparisons by Tukey’s post hoc test

### Inhibition of Either HDAC1 or miR-124-5p up-Regulates Neurotransmitter Expression in Depressed Rats

Depression was related to brain neurotransmitter disorders. Therefore, the levels of DA, NE, and 5-HT neurotransmitters in rat hippocampus were measured by ELISA. The results indicated that (Fig. 3b–d) with the normal group by contrast, reduced levels of DA, NE and 5-HT were found in rats of the CUMS group, sh-NC group, sh-HDAC1 group, anti-miR-NC group and anti-miR-124-5p group (all *P* < 0.05). No difference was witnessed in the neurotransmitter expression in the CUMS group, sh-NC group and anti-miR-NC group (all *P* > 0.05). Relative to the sh-NC and anti-miR-NC groups, DA, NE and 5-HT levels increased in rats of the sh-HDAC1 and anti-miR-124-5p groups (all *P* < 0.05), implying that down-regulation of HDAC1 or reduction of miR-124-5p could up-regulate the levels of DA, NE and 5-HT in the hippocampus of depressed rats.

The article "HDAC1-Mediated MicroRNA-124-5p Regulates NPY to Affect Learning and Memory Abilities in Rats with Depression" was retracted in 2023. Reasons: manipulated images; original data or images not available; unreliable results or conclusions; concerns about the images.

### Inhibition of Either HDAC1 or miR-124-5p Suppresses Oxidative Stress and Inflammation in Depressed Rats

Oxidative stress-related and inflammatory factor expression in serum were measured. With respect to the normal group, SOD and GSH activities were impaired, while MDA, IL-1β, TNF-α and NO levels were increased in the other depression model groups (all *P* < 0.05). SOD and GSH activities, and levels of MDA, IL-1β, TNF-α and NO among the CUMS group, sh-NC group and anti-miR-NC group showed no difference (all *P* > 0.05). In relation to the sh-NC group and anti-miR-NC group, an increase was noticed in the SOD and GSH activities and a decrease was observed in the MDA, IL-1β, TNF-α, and NO levels in the sh-HDAC1 group and anti-miR-124-5p group (all *P* < 0.05) (Fig. 4a–f), indicating that depletion of HDAC1 or down-regulation of miR-124-5p could alleviate oxidative stress and inflammation in depressed rats.

**Fig. 4:** Inhibition of either HDAC1 or miR-124-5p suppresses oxidative stress and inflammation in depressed rats. **a**–**c** Effect of inhibition of either HDAC1 or miR-124-5p on SOD, MDA and GSH concentration in serum of depressed rats; **d**–**f** Effect of inhibition of either HDAC1 or miR-124-5p on IL-1β, TNF-α, and NO concentration in serum of depressed rats; *n* = 10; a *P* < 0.05 compared with the normal group; b *P* < 0.05 compared with the sh-NC group; c *P* < 0.05 compared with the anti-miR-NC group. Comparisons among multiple groups were evaluated by one-way ANOVA, and pairwise comparisons by Tukey’s post hoc test

### HDAC1 Mediates miR-124-5p to Regulate NPY

RT-qPCR and western blot analysis were adopted for detection of HDAC1, miR-124-5p and NPY in the hippocampus. It was outlined that (Fig. 5a, b) versus the normal group, HDAC1 and miR-124-5p increased and NPY decreased in the CUMS group (all *P* < 0.05). HDAC1, miR-124-5p, and NPY expression showed no variations in the CUMS group and sh-NC group (all *P* > 0.05). Relative to the sh-NC group, the sh-HDAC1 group was reflected by decreased HDAC1 and miR-124-5p and elevated NPY expression levels (all *P* < 0.05). The above findings suggested the successful lentivirus interference and the positive relation between miR-124-5p and HDAC1 expression.

**Fig. 5:** HDAC1 mediates miR-124-5p to regulate NPY. **a** HDAC1, miR-124-5p and NPY mRNA expression in hippocampal tissues after inhibition of HDAC1 by RT-qPCR (*n* = 6); **b** HDAC1 and NPY protein expression in hippocampal tissues after inhibition of HDAC1 by western blot analysis (*n* = 6); **c** MiR-124-5p and NPY mRNA expression in hippocampal tissues after inhibition of miR-124-5p by RT-qPCR (*n* = 6); **d** NPY protein expression in hippocampal tissues after inhibition of miR-124-5p by western blot analysis (*n* = 6); a *P* < 0.05 compared with the normal group; c *P* < 0.05 compared with the sh-NC group. Comparisons among multiple groups were evaluated by one-way ANOVA, and pairwise comparisons by Tukey’s post hoc test

Also, miR-124-5p and NPY expression after miR-124-5p suppression were detected with the results (Fig. 5c, d) demonstrating that in relation to the normal group, elevated miR-124-5p and reduced NPY were presented in the CUMS group (both *P* < 0.05). On the contrary, the anti-miR-124-5p group trended toward decreased miR-124-5p and elevated NPY in relation to the anti-miR-NC group (both *P* < 0.05). No discrepancy was recognized in the miR-124-5p and NPY expression in the CUMS group and anti-miR-NC group (both *P* > 0.05). The results were indicative of the successful lentivirus interference and the negative connection between NPY and miR-124-5p.

The article "HDAC1-Mediated MicroRNA-124-5p Regulates NPY to Affect Learning and Memory Abilities in Rats with Depression" was retracted in 2023. Reasons: manipulated images; original data or images not available; unreliable results or conclusions; concerns about the images.

ChIP assay was to test whether HDAC1 could bind to the miR-124-5p promoter, and the results depicted that (Fig. 6a, b) HDAD1 was only related to the miR-124-5p promoter (*P* < 0.001), indicating that HDAC1 could directly regulate miR-124-5p.

**Fig. 6:** HDAC1 binds to the promoter of miR-124-5p. **a** Binding abundance of HDAC1 and miR-124-5p promoter region in HEK293T cells by ChIP assay (*n* = 3); **b** Binding abundance of HDAC1 and unrelated intergenic regions in HEK293T cells by ChIP assay (*n* = 3); **c** MiR-124-5p and NPY binding site by biological information software website; **d** Targeting relationship between miR-124-5p and NPY by dual luciferase reporter gene assay (*n* = 3); Comparisons between two groups were tested by *t* test

The targeting relationship between miR-124-5p and NPY was predicted and verified through RNA22 tool and dual luciferase reporter gene assay (Fig. 6c, d). With respect to the cells co-transfection with NPY-3′UTR-WT and mimic NC, the cells with co-transfection of NPY-3′UTR-WT and miR-124-5p mimic showed impaired luciferase activity (*P* < 0.05). No difference was recognized in the luciferase activity in the cells co-transfected with NPY-3′UTR-MUT and mimic NC, and the cells co-transfected with NPY-3′UTR-MUT and miR-124-5p mimic (*P* > 0.05).

### Knockdown of NPY Abolishes the Protective Effects of Inhibited miR-124-5p on Depressed Rats

Spontaneous depletion of NPY and miR-124-5p was programmed to explore their interplay in depressed rats. It was exhibited that (Fig. 7a, b) lower NPY expression level was noticed in the anti-miR-124-5p + sh-NPY group versus the anti-miR-124-5p + sh-NC group (*P* < 0.05). Body weight and behavioral function tests illustrated that (Fig. 7c–f) by comparison with the anti-miR-124-5p + sh-NC group, the rats in the anti-miR-124-5p + sh-NPY group presented reduced weight, SPP, frequency of crossing the grid, incidence of rearing and space exploration time with increased escape latency (all *P* < 0.05). HE staining of the hippocampal lesions pictured that (Fig. 8a) in comparison with the anti-miR-124-5p + sh-NC group, the number of hippocampal neurons was reduced, and hippocampal neurons were darkly stained, sparsely and disorderly arranged in an irregular shape with reduced cell layers in the anti-miR-124-5p + sh-NPY group. Moreover, versus the anti-miR-124-5p + sh-NC group, the rats in the anti-miR-124-5p + sh-NPY group was accompanied by reduced DA, NE and 5-HT (all *P* < 0.05) (Fig. 8b). Besides, impaired SOD and GSH activities, and increased MDA, IL-1β, TNF-α and NO levels existed in the rats of the anti-miR-124-5p + sh-NPY group versus the anti-miR-124-5p + sh-NC group (all *P* < 0.05) (Fig. 8c, d). Collectively, knockdown of NPY abolished the protective effects of repressed miR-124-5p on depressed rat.

The article "HDAC1-Mediated MicroRNA-124-5p Regulates NPY to Affect Learning and Memory Abilities in Rats with Depression" was retracted in 2023. Reasons: manipulated images; original data or images not available; unreliable results or conclusions; concerns about the images.

**Fig. 7:** Knockdown of NPY abolishes the effects of inhibited miR-124-5p on body weight and behavioral function of depressed rats. **a** MiR-124-5p and NPY mRNA expression in hippocampal tissues after inhibition of both miR-124-5p and NPY by RT-qPCR (*n* = 6); **b** NPY protein expression in hippocampal tissues after inhibition of both miR-124-5p and NPY by western blot analysis (*n* = 6); **c** Body weight of depressed rats after inhibition of both miR-124-5p and NPY (*n *= 10); **d** SPP of depressed rats after inhibition of both miR-124-5p and NPY (*n* = 10); **e** Frequency of crossing the grid and incidence of rearing after inhibition of both miR-124-5p and NPY (*n* = 10); **f** Escape latency and space exploration time after inhibition of both miR-124-5p and NPY (*n* = 10); Comparisons between two groups were tested by *t* test

**Fig. 8:** Knockdown of NPY abolishes the effects of inhibited miR-124-5p on hippocampal damages of depressed rats. **a** HE staining of hippocampal lesions of rats after inhibition of both miR-124-5p and NPY (*n* = 6); **b** ELISA of NE, 5-HT and DA expression in hippocampal tissues of rats after inhibition of both miR-124-5p and NPY (*n* = 6); C. Effect of inhibited NPY and suppressed miR-124-5p on SOD, MDA and GSH concentration in serum (*n* = 10); D. Effect of inhibited NPY and suppressed miR-124-5p on IL-1β, TNF-α and NO concentration in serum (*n* = 10). Comparisons between two groups were tested by *t* test

The article "HDAC1-Mediated MicroRNA-124-5p Regulates NPY to Affect Learning and Memory Abilities in Rats with Depression" was retracted in 2023. Reasons: manipulated images; original data or images not available; unreliable results or conclusions; concerns about the images.

## Discussion

Depression is a type of psychiatric disorder comprising a variety of conditions with diverse symptoms [20]. Though emerging studies have implied the role of miRNAs in depression, the precise action of miR-124-5p has been rarely investigated. Hence, the present study is projected for better comprehension of the mechanism of miR-124-5p/HDAC1/NPY axis in depression with the major outcome elaborating that silencing of either HDAC1 or miR-124-5p up-regulated NPY to improve memory and learning abilities of depressed rats.

To begin with, this study discovered HDAC1 expression in hippocampal tissues with the findings suggesting the elevation in the HDAC1 expression. Subsequently, with the purpose to decipher the functional roles of HDAC1 in depressed rats, loss-of-function assays were performed and it was disclosed that knockdown of HDAC1 increased the body weight, improved learning and memory abilities, attenuated pathological damage, up-regulated neurotransmitter expression, and suppressed oxidative stress and inflammation in depressed rats. Currently, a study has implied an increment in the expression of HDAC1 in depressive-like and anxiety-like phenotypes resulted by stress-offspring [21]. Moreover, the expression of HDAC1 is documented to up-regulate in penumbra in photothrombotic stroke [22]. Besides that, the incremental HDAC1 mRNA expression is found in granule and pyramidal cells in temporal lobe epilepsy [23]. As to the functional role of HDAC1, it has been reported that virus-mediated overexpression of neuronal HDAC1 in the hippocampus of mice imposes influences on loss of contextual fear memory in particular [24]. Mechanically, HDAC inhibitors reverse cognitive deficits found in neurodegenerative diseases and age-related memory loss [25]. Actually, it is accepted that the HDAC1 suppression by tianeptinaline has advanced neuroplasticity and reinforced memory [26]. As mentioned in a prior study, it is concluded that repression of HDAC1 inhibits the pathogenic processes that lead to motor neuron degeneration in mitochondrial diseases [27]. Experimentally, the silencing of HDAC1 by 5-thienyl-substituted 2-aminobenzamide-type is partially involved in the prevention of neuronal cell death in Parkinson's disease models [28]. Further supported by those researches, the protective effects of silenced HDAC1 have been witnessed in brain diseases, including but not limited to depression.

Then, our study discovered a targeting relationship between HDAC1 and miR-124-5p, which was supported by a prior study which suggests miR-124 transcription is in the charge of EVI1, acting by connection with the deacetylase HDAC1 [29]. miR-124-5p was the overexpressed gene in depressed rats and knockdown of miR-124-5p had the similar functions of silenced HDAC1 in depressed rats. In fact, there is a study indicating that the expression of miR-124 in the hippocampus is up-regulated from 5 to 6 weeks in depression-like behavior phenotypes [7]. Another study has identified the increase in the miR-124 expression in female with cocaine use disorder [30]. Also, it is previously described that miR-124-3p is highly expressed in stressed rodents in major depressive disorder [31]. Regarding to the effects, knockdown of miR-124 in the prefrontal cortex is reported to attenuate depression-like behavior of mice [9]. Besides that, miR-124 knockdown is believed to serve as an antidepressant agent of chronic corticosterone-induced gypenosides in mice [32]. Drawn from a prior study, knockdown of miR-124 can result in improved behavioral susceptibility to a milder stress paradigm [33]. It is reported that suppression of miR-124 by lentivirus transfection in the hippocampus can protect ketamine-induced neurodegeneration in vivo and in vitro [34]. Anyway, miR-124-5p suppression is an active actor to attenuate depression.

The article "HDAC1-Mediated MicroRNA-124-5p Regulates NPY to Affect Learning and Memory Abilities in Rats with Depression" was retracted in 2023. Reasons: manipulated images; original data or images not available; unreliable results or conclusions; concerns about the images.

Furthermore, NPY expression was verified to be regulated by HDAC1 and miR-124-5p. The deteriorated deficits associated with HDAC2 in histone acetylation may be related to the decreased expression of NPY and can used to control anxiety-like and drinking behaviors [14]. NPY was down-regulated in depressed rats and up-regulation of NPY promoted learning and memory ability recovery in depressed rats. In the development of depressive-like behaviors, the rat models are manifested with reduced NPY expression [17]. Academically, the expression of NPY is evidenced to decline in mice with depression [35]. Consistently, the above-mentioned study findings are as same as the previous literature to some extent.

The novel findings of study suggested that inhibited miR-124-5p or suppressed HDAC1 attenuated learning and memory abilities and increased body weight of depressed rats. In addition, knockdown of miR-124-5p or inhibition of HDAC1 suppressed oxidative stress and inflammation and promoted neurotransmitter expression of depressed rats. Moreover, HDAC1 mediated miR-124-5p to regulate NPY. In the rescue experiments, knockdown of NPY abolished the protective effects of inhibited miR-124-5p on depressed rats.

## Conclusion

In summary, this study highlighted the effect of HDAC1/miR-124-5p/NPY axis in depression with the major findings suggesting inhibited miR-124-5p or suppressed HDAC1 attenuated learning and memory abilities, increased body weight, suppressed oxidative stress and inflammation, as well as promoted neurotransmitter expression in depressed rats. HDAC1/miR-124-5p/NPY axis may provide a reference to treat neurological disorder, which may also update the existed knowledge of depression. However, further studies are still required for thorough comprehension of the complex mechanism of HDAC1/miR-124-5p/NPY axis in depression.

The article "HDAC1-Mediated MicroRNA-124-5p Regulates NPY to Affect Learning and Memory Abilities in Rats with Depression" was retracted in 2023. Reasons: manipulated images; original data or images not available; unreliable results or conclusions; concerns about the images.

## Data Availability

Not applicable.

## Abbreviations

miR-124-5p: MicroRNA-124-5p
HDAC1: Histone deacetylase 1
NPY: Neuropeptide Y
CUMS: Chronic unpredictable mild stress
SD: Sprague–Dawley
SPF: Specific pathogen-free
NC: Negative control
OFT: Open field test
SPT: Sucrose preference test
SPP: Sucrose preference percentage
MWM: Morris water maze test
SOD: Superoxide dismutase
MDA: Malondialchehyche
GSH: Glutathione
IL-β: Interleukin-β
TNF-α: Tumor necrosis factor-α
NO: Nitric oxide
ELISA: Enzyme-linked immunosorbent assay
HE: Hematoxylin–eosin
BCA: Bicinchoninic acid
NE: Norepinephrine
5-HT: Serotonin
DA: Dopamine
RT-qPCR: Reverse transcription quantitative polymerase chain reaction
cDNA: Complementary DNA
SDS: Sodium dodecyl sulfate
ChIP: Chromatin immunoprecipitation
UTR: Untranslated region
MUT: Mutant type
WT: Wild type
ANOVA: One-way analysis of variance
